The article "Efficacy of Enhanced Cytokine-Induced Killer Cells as an Adjuvant Immunotherapy for Renal Cell Carcinoma: Preclinical and Clinical Studies" was published in 2021. Journal: J Healthc Eng.

# Efficacy of Enhanced Cytokine-Induced Killer Cells as an Adjuvant Immunotherapy for Renal Cell Carcinoma: Preclinical and Clinical Studies

**DOI:** 10.1155/2021/5709104

**Published:** 2021-09-08

**Authors:** Yang Yang, Run-Qing Wang, Yi-Ming Zhong, Ming-Yao Meng, Yi-Yi Zhao, Li-Rong Yang, Lin Li, Zong-Liu Hou

**Affiliations:** ^1^Central Laboratory of Yan'an Hospital Affiliated to Kunming Medical University, Kunming, Yunnan Province, China; ^2^Key Laboratory of Tumor Immunological Prevention and Treatment of Yunnan Province, Kunming, Yunnan Province, China; ^3^Kunming Medical University, Kunming, Yunnan Province, China; ^4^Yunnan Cell Biology and Clinical Translation Research Center, Kunming, Yunnan Province, China

## Abstract

Cytokine-induced killer (CIK) cells have been proved to be an effective method of tumor immunotherapy in numerous preclinical and clinical studies. In our previous study, a new method was developed to prime and propagate CIK cells by the combination of IL-2 and IL-15, and this kind of CIK cells had enhanced antitumor effect on lung cancer. For renal cell carcinoma (RCC), immunotherapy plays an important role because of the poor efficacy of radiotherapy and chemotherapy. In this study, we further evaluated the antitumor effects of these enhanced CIK cells against RCC. Enhanced CIK cells were generated by IL-2 combined with IL-15 and identified by flow cytometry. HEK-293 and ACHN cell lines were used to verify the efficiency of CIK cells *in vitro*, and then the ACHN tumor xenograft model was also employed for *in vivo* study. In addition, the secreted cytokines including IFN-*γ*, granzyme B, TNF-*α*, and perforin, as well as the local microstructure were also studied. Subsequently, 20 patients with RCC were enrolled into our study, and 11 patients were randomly divided into the autologous CIK treatment group for clinical research. The results showed that enhanced CIK cells exert better antitumor effects in RCC *in vitro* (*p* < 0.01 in HEK-293 and *p* < 0.05 in ACHN）and *in vivo* (*p* < 0.05). Patients benefit overall survival from enhanced CIK therapy in our clinical study. Our present preclinical and clinical studies for the first time elucidated that these enhanced CIK cells would be used as an effective adjuvant therapy in the treatment of RCC.

## 1. Introduction

Renal cell carcinoma (RCC) is the most common malignant tumor of adult kidney and the third common malignancy in the urological system, accounting for more than 2% of all tumors [1]. In 2018, new cases of RCC worldwide were estimated to be 403, 262, which led to more than 175,000 deaths [2, 3]. Surgical resection, including partial nephrectomy and radical nephrectomy, is the gold standard treatment of localized RCC. Nevertheless, up to 30% of RCC cases had metastasized at the time of diagnosis [2]. In addition, the local recurrence rate of RCC after surgical treatment is close to 20%–30% within 3 years [4]. With unique biological characteristics, RCC shows poor response on traditional nonoperative treatment such as radiotherapy and chemotherapy. The overall effective rate of chemotherapy on RCC is less than 5-6%, and the radiotherapy is even worse [5]. Immunotherapy based on IL-2 and IFN-*α* was the main adjuvant therapy before the adoptive cell-mediated immunotherapies, and targeted immunotherapies were used for metastatic renal cell cancer (MRCC). Although IL-2 and IFN-*α* were recommended as a first-line treatment in the past 20 years, they could hardly improve the survival [6–8].

In the past decades, adoptive cell immunotherapies developed rapidly and played more and more important roles in tumor immunotherapy. The CIK cells, a group of heterogeneous immune cells stimulated by cytokines, showed notable antitumor cytotoxic activities *in vitro* and *in vivo* on malignant tumors. The conventional CIK cells used in numerous studies were generated from peripheral blood mononuclear cells (PBMCs) with the addition of IFN-*γ*, anti-CD3 antibodies, and IL-2 [9, 10]. The cytokines IFN-*γ* and IL-2 are crucially involved in the cytotoxicities of the CIK cells, and anti-CD3 antibodies provide a mitogenic signal to T cells for proliferation [11]. However, since 2010, we developed the new stimulation method to induce enhanced CIK cells, which were primed and propagated with IL-2 and IL-15. IL-15 has a function similar to IL-2, which can effectively promote the activation, proliferation, and long-term survival of T cells and NK cells [12]. More than this, as the maintenance factor of CD8+ memory T cells, IL-15 can activate CD44hiCD8+ T cells selectively and promote T cells transform into memory T cells [13]. Our previous studies found these enhanced CIK cells possessed stronger antitumor activities on lung adenocarcinoma compared with conventional CIK cells [14]. Other previous studies showed conventional CIK cells could ameliorate the prognosis of inoperable RCC patients and extend the survival of those patients after nephrectomy [15]. Therefore, in this present study, the effects of our enhanced CIK cells on RCC would be also evaluated *in vitro* and *in vivo*. Meantime, the eligible patients with RCC were enrolled into our study and treated with enhanced CIK cells. The safety and efficacy of these cells were also further assessed. These enhanced CIK cells were comprehensively researched on RCC in this study, and it is shown that these enhanced CIK cells can be an effective choice in RCC immunotherapy.

## 2. Materials and Methods

### 2.1. Cell Lines, Animal, and Reagents

Human renal cell carcinoma cell lines HEK-293 and ACHN were obtained from Cell Cook (Guangdong, China). Both of them were incubated at 37°C in a 5% CO_2_, 95% humidified atmosphere with RPMI 1640 growth medium. Cytokines for CIK cell production, including IL-2, IL-15, and IFN-*γ* were from Pepro Tech. The CD3 monoclonal antibody OKT3 (MACS GMP CD3 pure) was from Miltenyi Biotech, Germany. The fluorescence-conjugated antibodies against Ki-67 and CD3 were purchased from BD Biosciences (San Jose, USA) and R&D Systems (Minneapolis, USA). The cell proliferation assay kit was Cell Counting Kit-8 (Dojindo Molecular Technologies, Rockville, USA). The ELISA kits for measurement of human TNF-*α*, IFN-*γ*, perforin, and granzyme B were obtained from Neo Bio Science (Beijing, China). Gluta electron microscope fixative was obtained from Solarbio (Beijing, China). The TUNEL assay kit was purchased from Roche (Basel, Switzerland).

### 2.2. Preparation of Enhanced CIK Cells and Flow Cytometry

The use of fresh human buffy coat was approved by the ethics committee of Yan'an Hospital of Kunming Medical University. The CIK cells were derived from PBMCs. PBMCs were cultured in RPMI 1640 growth medium which contained 10% FBS, 100 U/ml penicillin, 2% L-glutamine, and 10 U/ml streptomycin at a density of 1 × 10^6^ cells/ml. The generation of enhanced CIK cells was induced by adding 1,000 U/mL IFN-*γ* on day 0 and 100 ng/mL OKT3, 500 U/mL IL-2, and 10 ng/mL IL-15 within the following 24 h of culture. The CIK cells were stimulated with 500 U/mL IL-2 and 10 ng/mL IL-15 every 5 days. The enhanced CIK cells were cultured for 15 days, and their phenotypes were analyzed. At the same time, another group of CIK cells were dealt without IL-15 for control. The proliferation rate of these two kinds of CIK cells was detected and compared on the 7^th^, 9^th^, 11^th^, 13^th^, and 15^th^ day.

The expression of surface markers of CIK cells, such as CD3, CD4, CD8, and CD56 (BD Biosciences), was monitored by flow cytometry at day 15. In brief, the enhanced CIK cells were harvested by centrifugation at a speed of 2000 ×g. The cell pellets were suspended with blocking buffer. After washing with blocking buffer, the cells were stained with corresponding mAbs for 30 min at room temperature. After staining, the cells were washed twice, then examined by Beckman Coulter Gallios Flow Cytometry system, and the data were analyzed by FlowJo software.

### 2.3. Cytotoxicity Assay

The cytotoxic effects of CIK and enhanced CIK cells on ACHN cells and HEK-293 cells were investigated by Cell Counting Kit-8-based assay. At the same time, we used other four cell lines including SPC-A-1 (human lung adenocarcinoma cell line), HCT-116 (human colorectal cancer cell line), BGC 823 (human gastric cancer cell line), and BEL 7404 (human hepatoma cell line) as the nonkidney cell lines for control. Each kind of target cells (at 5 × 10^3^ cells/well) was seeded into a 96-well plate for 24 h. Then, the two kinds of CIK cells were incubated with the target cells at ratio of 8 : 1, 16 : 1, 32 : 1, and 64 : 1 (effector cell/target cell). The target cells without any treatment were taken as control. After 36 h, the supernatants including CIK cells in the wells were aspirated completely and then washed with PBS gently. CCK-8 solution and fresh-cultured medium were added into each well, and the samples were incubated at 37°C for 2 h. The absorbance was measured at 450 nm using a microplate spectrophotometer (Varioskan Lux, Thermo Scientific, USA). The cell viability was calculated according to the following formula: cell viability (%) = ((*E* − *B*)/(*N* − *B*))100, where *E* is the experimental CCK8 release in effector plus target cell cocultures, *B* is the spontaneous release by medium alone, and *N* is the spontaneous release by target cells alone. Three independent samples with triplicated wells were measured, and the mean value was calculated.

### 2.4. Scanning Electron Microscopy

1 × 10^6^ ACHN cells were seeded in the culture dishes (100 mm^2^). After tumor cells attachment, 8 × 10^6^ enhanced CIK cells were incubated with ACHN cells. All cells were harvested from plates by gently scraping after 36 h of treatment and subsequently suspension-fixed in glutaraldehyde for 24 h at 4°C and rinsed with cold PBS for 3 times. The samples were dehydrated by ethanol gradient (50% to absolute ethanol, each for 15 min) and soaked in isoamyl acetate/ethanol mixture (1 : 1, v/v). The samples were gold-sputtered after prepared by the CO_2_ critical point dry and then examined through a scanning electron microscope (Nova NanoSEM 450, FEI, Czech Republic).

### 2.5. Tumor Xenograft Model

Four-week-old male BALB/c nude mice were provided by SJA Laboratory Animal Co. (Hunan, China). The procedures of animal experiment complied with the National Institutes of Health Guidelines for the Care and Use of Laboratory Animals. The animal studies and protocol were approved by the Experimental Animal Ethics Committee of Yan'an Hospital of Kunming Medical University. All surgeries were performed under anesthesia, and all efforts were made to minimize the suffering. 3 × 10^6^ ACHN cells/mouse were suspended in 200 *μ*L PBS and injected subcutaneously into the backs of the BALB/c nude mice. The tumor formation was monitored after injection by time. Tumor volume was measured weekly with a caliper and calculated using the formula length × width^2^/2. When the tumor volumes reached 0.2 cm^3^, the mice were divided into four groups randomly. They were PBS intratumoral injection group, CIK intratumoral injection group, PBS intravenous injection group, and CIK intravenous injection group (9 mice each). The treatments were conducted on the 14^th^ day after tumor inoculation. 2 × 10^7^ enhanced CIK cells per mouse were suspended in 200 *μ*L saline and injected intratumorally or intravenously through the tail vein once a week. The CIK treatments were administered for 3 times. In control groups (both PBS intratumoral injection group and PBS intravenous injection group), 200 *μ*L saline was injected for each mouse instead of CIK cells. On day 35, the mice were anesthetized with sodium pentobarbital (10 mg/kg) and sacrificed. Then, the tumors were excised and fixed with 4% paraformaldehyde after weighted. Blood from mice was centrifuged, and the serum was stored at −80°C for further analysis.

### 2.6. ELISA Assay of Cytokines

ACHN cells or HEK-293 cells (both 3 × 10^4^ cells/well) were seeded in 6-well plates, and then 9.6 × 10^5^ CIK cells were added into the wells. The supernatant of ACHN cells or HEK-293 cells cocultured with CIK cells for 36 h were collected. The supernatant samples of cells were analyzed with an enzyme-linked immunosorbent assay (ELISA) kit for IFN-*γ*, perforin, TNF-*α*, and granzyme B (Neo Bio Science, Beijing, China). Additionally, the expressions of above proteins in the serum from each mouse which was administrated with enhanced CIK or PBS were also detected by ELISA. The protein expression levels were measured according to the manufacturer's instructions.

### 2.7. Immunofluorescence Assay

After fixation for 7 days, the tumor tissues were dehydrated and embedded in paraffin. The samples were sectioned in paraffin (5 *μ*m) by a sliding microtome, and the tissue sections were heated at 56°C for 48 h. Then, the slides were deparaffinized and rehydrated into EDTA buffer (pH 8.0) for antigen retrieval. The slides were incubated with primary antibodies against CD3 (human), Ki-67, and TUNEL reaction mixture overnight at 4°C, after 3% BSA was used to block nonspecific binding for 30 min. On the following day, the sections were incubated with secondary antibody, at room temperature for 50 min in dark. DAPI solution was used for counterstain. The positive expression of CD3, Ki-67, and the DNA strand breaks during apoptosis (TUNEL) was observed and captured under a fluorescent microscope (Nikon Eclipse C1, Japan). Five captures were selected randomly from each slice, and the number of positive-stained cells was counted by Image-Pro Plus 6.0. The data expressed as the percentage of positive-stained cells were analyzed by GraphPad Prism 7.

### 2.8. Clinical Study

Twenty RCC patients in the urology department of Yan'an Hospital affiliated to Kunming Medical University from 2011 to 2014 were enrolled in this study. Partial nephrectomy or radical nephrectomy was performed to all patients, and RCC was diagnosed and confirmed by pathological examination. Among these patients, 11 subjects were treated with autologous CIK cells. Meantime, another 9 subjects were enrolled as controls, and no adjuvant therapy was conducted except for two patients with metastasis. These two patients received immunotherapy of IL-2 and IFN-*α*. This study was approved by the Ethics Committee of Yan'an Hospital of Kunming Medical University, Yunnan, China, complied with the guidelines of the Declaration of Helsinki. Informed consent was obtained from all subjects before they enrolled into the study. The treatment schedule for the study consisted of 3 to 5 cycles of enhanced CIK cell infusions, and each cycle included 3 infusions in 1 week and followed by a three-week rest. PBMCs were isolated from patients with RCC and cultured with IFN-*γ*, OKT3, IL-2, and IL-15 according to the above methods. After 14 days, CIK cells were gathered and analyzed for phenotype. All cell products were detected to be free of mycoplasma, bacterial, and fungal contamination. Patients received about 1.5 × 10^7^ autologous CIK cells/kg for each infusion. All patients were followed up every 3 months during 2 years and then every 6 months until they were died, lost contact, or end follow-up on December 31, 2017. Tumors were assessed every 2 months by using the Response Evaluation Criteria in Solid Tumors (RECIST) guidelines since the first CIK treatment. Tumor responses were reported as complete responses (CR), partial responses (PR), stable disease (SD), or progressive disease (PD). All subjects were monitored for local and systemic toxicity before, during, and after treatment.

### 2.9. Statistical Analysis

All data were analyzed with GraphPad Prism 7 statistical software. The values were expressed as means ± S.D. (or S.E.M.). Statistical data were analyzed by Student's *t*-tests. *p* < 0.05 was considered to be statistically significant. The overall survival (OS) and progression-free survival (PFS) were evaluated by Kaplan–Meier analysis.

## 3. Results

### 3.1. The Proliferation Rate and Phenotypic Analysis of Enhanced CIK Cells Expanded with IL-2 and IL-15

The proliferation rate of enhanced CIK cells was higher than that of CIK cells from the thirteenth day significantly (Figure 1(c)). Flow cytometry was used to detect the immunophenotypes of CIK cells and enhanced CIK cells. The results showed that the proportion of CD3+, CD3+CD4+, CD3+CD8+, and CD3+ CD56+ was obviously increased in both CIK cells compared with the corresponding PBMC after expanding for 15 days (Figure 1(a)). Furthermore, the proportion of CD3+ CD56+ in enhanced CIK cells was obviously higher than that in conventional CIK cells. The difference between each subset was statistically significant (*p* < 0.001, Figure 1(b)).

### 3.2. Cytotoxicities of Enhanced CIK Cells against Tumor Cells

The cell viabilities of ACHN cells, HEK-293 cells, SPC-A-1 cells, HCT-116 cells, BGC 823 cells, and BEL 7404 cells incubated with conventional CIK and enhanced CIK cells for 36 h are shown in Figure 2. The curves of RCC cell viability at different ratios showed that both CIK cells significantly killed HEK-293 and ACHN cells at an *E*/*T* ratio of 8 : 1, 16 : 1, 32 : 1, and 64 : 1, and the enhanced CIK cells showed higher efficiency to kill the RCC cells at the high *E*/*T* ratio (Figure 2(a)). The median cell viabilities of HEK-293 and ACHN cells after incubation with enhanced CIK cells at an *E*/*T* ratio of 64 : 1 were 25.9% and 20.5%, respectively (Figure 2(a)). The cytotoxicities of enhanced CIK cells showed dose-effect relation on tumor cells. Meanwhile, the nonkidney cells showed two different responses after CIK cell incubation. Enhanced CIK cells inhibited SPC-A-1 and HCT-116 cancer cell growth more effectively than conventional CIK cells. However, the difference effects between enhanced and conventional CIK cells on BEL-7407 and BCG-823 cells were not obvious.

### 3.3. Cytokines Induced by CIK Cells after Coculture with Tumor Cells

The levels of granzyme B (GrzB), perforin, TNF-*α*, and IFN-*γ* from the supernate of ACHN cells/HEK-293 cells incubated with conventional CIK and enhanced CIK cells for 36 h, were detected by ELISA. As shown in Figure 2(b), the levels of GrzB, TNF-*α*, and IFN-*γ* in ACHN + enhanced CIK group and HEK-293+enhanced CIK group were significantly increased compared with the conventional CIK group, while the inductive effect on perforin level was relatively mild which was not significantly different from the conventional CIK group.

### 3.4. The Interaction between CIK Cells and Tumor Cells under Electron Microscopy

As shown in Figure 3, the CIK cells enclosed ACHN cells with their pseudopods and adhered to tumor cells tightly under a scanning electron microscope at 2500x, 5000x, 14000x, and 30000x magnification, respectively. The CIK cells were much smaller and rounder compared with the renal carcinoma cells ACHN through the morphological observation.

### 3.5. The Antitumor Abilities of Enhanced CIK Cells in ACHN Human Renal Tumor Xenografts

Since enhanced CIK cells showed promising results on *in vitro* studies, further animal studies were carried out. The xenograft model of BALB/C nude mice with ACHN cells was successfully established and employed in this study. The results showed that the tumor weights were significantly reduced after enhanced CIK injection both through tail vein and intratumoral (Figures 4(a) and 4(b)). Especially, the suppressive effect of CIK via administration intravenously was stronger than that of CIK through administration intratumorally. Tumor weight in the intravenous injection group was found to decrease by 56.9% vs. control group; however, it just reduced by 30.2% in the intratumoral injection group. And, no significant differences between CIK treatment groups and control groups were observed in body weight (Figure 4(c)). In addition, the levels of granzyme B, perforin, and IFN-*γ* in serum from mice were more or less increased after CIK treatment compared with the control, although there was no significant difference (Figures 4(d)–4(f)). Meanwhile, the tumors collected from different treatment groups were subject to immunofluorescence staining. Among the tumor sections stained with TUNEL, the number of apoptotic cells was significantly higher in the CIK-treated group than those in the PBS control group (Figures 5(a) and 5(c)). In addition, the number of Ki-67 positive-stained cells in tumor sections was significantly lowered in the CIK treatment group than that in PBS group (Figures 5(a) and 5(c)). To further confirm CIK cells in the intravenous injection group which could migrate and reside in tumor sites, the CD3 positive-stained cells which represented CIK cells were also analyzed by immunofluorescence staining. When compared with the control group, the number of CD3 positive-stained cells in tumor samples is higher following CIK intravenous treatment (Figures 5(b) and 5(c)). The above results indicated that the antitumor effects of CIK cells were associated with induction of apoptosis and reduction of proliferation of tumor cells.

### 3.6. Patient Outcomes

In view of enhanced CIK cells showing effective antitumor activities on RCC without obvious side effect through the preclinical evaluation, the therapeutic benefit of these cells was further assessed in patients with RCC after the partial nephrectomy or radical nephrectomy. The demographics and clinical characteristics of the patients in both control group and CIK group are listed in Tables 1 and 2, and there were no significant differences on age/sex and TMN staging between two groups. No obvious adverse reactions occurred except two patients with slight fever, one patient with few rashes, and one patient with muscular soreness after CIK administration. In addition, these reactions were all disappeared within few hours. The overall condition of patients was improved after CIK cell treatment including mental state and physical condition. The median follow-up period was 45 months. Five patients (45%) in the CIK group showed a complete response, and 4 patients (36%) showed stable disease (Table 1). The lung metastasis in RCC patients was not lessened after CIK treatment, but the state of metastasis was stable during follow-up. The representative CT scan images showed that ung metastasis in one patient had tardy progress in 60 months, and the metastatic lesions in another patient remained unchanged in 18 months (Figure 6(b)). In the control group, there were 2 complete responders (22%), and 4 patients (44%) had disease stabilization. Meanwhile, 3 patients (33%) had continuous disease progression, and one patient (case6) died of rapid exacerbation of lung metastasis (Table 2). The overall survival (OS, log-rank, *p*=0.0470) in the CIK group was longer than that in the control group significantly. The median OS in the CIK group was 45 months (vs. 29 months in control) during follow-up. However, there were no significant differences of progression-free survival (PFS) between the two groups (log-rank, *p*=0.2012) (Figure 6(a)). At the end of follow-up, two patients were dead. One of them died of heart disease who was from the CIK group (case 6), and the other one died of lung metastasis who was from the control group (case 6).

## 4. Discussion

Renal cell carcinoma (RCC) is one of the ten most common malignant tumors in adults, but it shows very different characteristics from other tumors [5]. Due to its resistance to radiotherapy and chemotherapy, the potential treatment option has focused on immunotherapy as the adjuvant treatment of RCC. CIK cells, an immunotherapy highly applied in various malignant tumors, has also been used in the treatment of RCC in the past decade [15, 16]. In the previous study of our department, the enhanced CIK cells stimulated with IL-2 and IL-15 had shown better proliferative potential than conventional CIK cells [11]. We analyzed the proliferation curve of enhanced CIK cells and confirmed that the proliferation rate of enhanced CIK was more than twice that of conventional CIK. High yield of enhanced CIK cells can reduce the demand of autologous peripheral blood and more efficiently in clinical CIK treatment. Although the *ex vivo* protocols for the production of CIK cells are distinct, CIK cells mainly consisted of CD3^+^CD56^−^ T cells, CD3^−^ CD56^+^ NK cells, and CD3^+^CD56^+^ NKT cells, and the major effector cells were CD3^+^CD56^+^ T cells [17]. According to several studies of CIK cells, the proportion of CD3+CD56+ NKT-like cells was 20%–60% [15, 18, 19]. Then, the data of flow cytometry showed that our enhanced CIK cells were also heterogeneous cells mass and a majority of CD3+CD56+ NKT-like cells, and the average proportion of these subsets was more than 80%, better than conventional CIK cells.

The intrinsic mechanism of the antitumor effect in CIK cells has been continuously studied and explored. And, in our previous studies, we found NKG2D, FasL, and perforin/granzyme etc., of enhanced CIK cells which activated with IL-15, and IL-2 was significantly different compared with those of conventional CIK cells [20]. CIK's antitumor effect is mediated by various mechanisms such as several receptors FasL, NKG2D, TRAIL, and granzyme or perforin secretion [17]. In this present study, RCC cells treated with enhanced CIK cells also markedly induced the IFN-*γ* and perforin/granzyme secretion, which led to eradicate RCC cells through apoptosis. In addition, we also found some phenomena suggesting that CIK cells may have some unknown mechanism in the interaction with tumor cells. Referring to past studies, CIK cells killed tumor cells by MHC (major histocompatibility complex) unrestricted cytotoxicities, and the major effectors are cytokines [21].We observed that enhanced CIK cells surround and adhere to the surface of tumor cells, and there were pseudopodia-like structures between them (Figure 3). The view of immunofluorescence also showed that the enhanced CIK cells infiltrate and adhere to tumor cells (Figure 5(b)). In some studies, CIK cells were found to involve MHC-restricted manner by TCR engagement too, CIK cells trigger cellular immunity through this two mechanisms and exert dual antitumor effects, and it has both cytokine effect and MHC-restricted contact effect [22, 23].

Although CIK therapy was usually through intravenous administration clinically, intratumoral injection was also used in cancer treatment recently, especially the application of DC cells or tumor vaccine [24, 25]. Hence, in this study, two administration methods, intravenous injection and intratumoral injection was employed to evaluate the antitumor activities of enhanced CIK cells on RCC. Interestingly enough, our study showed the enhanced CIK cells significantly suppressed the growth of ACHN renal tumor xenografts by both of two administration methods, even more suppressive effect by intravenous injection of CIK cells. The most probable cause was the tumor microenviroment would affect the tumoricidal function of T cells or NK cells. Previous study demonstrated that intratumoral NK cells had reduced proliferative ability, decreased expression of activating receptors, and increased inhibitory receptors [26]. And, suppressive factors in tumor such as Treg, macrophage, and soluble mediators, for example, interleukin- (IL-) 10 and TGF-*β*, could impair cytotoxic function of CD8^+^ T cells [27]. Therefore, the injection of CIK cells directly into tumor might limit the activity of them. Meanwhile, intravenous injection of CIK cells did not diminish their ability and vitality at first time and subsequently induced intratumoral CD3+ lymphocyte infiltration (Figure 5(b)). Furthermore, intravenous administration of CIK cells showed the systemic effects of a boosting cellular immunity. The levels of CD3^+^CD8^+^, CD3^+^CD45RO^+^, and CD3^+^CD56^+^ cell amount and IFN-*γ* in patients' blood increased and lasted for half a year at least after CIK cells transfusion [28]. Zhang et al. also found that the ratio of CD3^+^ CD56^+^ T cells and CD3^+^ CD8^+^ T cells in peripheral blood of patients was still higher than that of the control group for a long time after CIK treatment [29]. CIK cells not only play a direct antitumor role, but also activate the host's immune system, maintaining a high proportion of CD3^+^ CD8^+^ T cells and CD3^+^ CD56^+^ T cells for a certain period of time, driving a sustained antitumor effect. Therefore, one of the possible reasons why intravenous injection of CIK cells showed stronger inhibitory effects on tumor growth than intratumoral injection which might be due to the higher population of CD3^+^CD56^+^ cells and even the memory cells existing in circulation. Of course, if the adoptive cell immunotherapy including CIK cells want to be applied in clinical better, the distribution and elimination of cell products, especially through different routes of administration, should be further investigated.

A systematic meta-analysis for seven selected trials which were conducted in 385 patients with RCC found adjuvant immunotherapy with CIK cells possessed certain efficacy and safety [30].The above results were consistent with our study. We observed that CIK cells can prolong the OS of RCC patients, and the median OS in the CIK cell therapy group was 45 months (vs. 29 months in control). However, there were only 20 subjects enrolled in the present study. More eligible patients should be included in future. In many clinical trials of CIK treatment in RCC, although the tumor could not completely disappear, the survival time of the patients with RCC was prolonged [15, 16, 31]. There were similar results in our clinical data, in enhanced CIK treatment, and the two RCC patients with lung metastasis were relatively stable and the lung lesions progressed slowly.

Taken together, for the first time, the present study demonstrated that the enhanced CIK cells activated by IL-2 and IL-15 exerted stronger antitumor effects on RCC *in vitro* and *in vivo* through IFN-*γ* and perforin/granzyme-induced apoptosis. The enhanced CIK cell treatment could provide a significant survival benefit to RCC patients (OS, *p*=0.0470), improve partial response rate, and have stable disease without serious adverse reactions. Of course, as a nonspecific tumor immunotherapy, CIK cells cannot completely remove tumor cells, and it has a mild but sustained antitumor effect. In the latest reports, CIK cells combined with PD-1 antibody and CTLA-4 antibody have achieved significant effect in the treatment of RCC [19, 32, 33].Additionally, it reported that CIK cells could enhance the antitumor activity of CAR-T cells [34]. After combination with sorafenib or sunitinib, CIK cells could effectively improve the OS and PFS of patients with metastatic RCC [35]. Especially, some studies indicated that this synergistic effect of CIK with other immunotherapy mainly depends on the CD3^+^CD56^+^ cells [36, 37]. Therefore, our enhanced CIK cells with a high proportion of CD3^+^CD56^+^ cells should be further studied and taken wider applications.

## 5. Conclusion

The enhanced CIK immunotherapy showed mild and long-lasting antitumor effect with satiety, although it can hardly remove the RCC thoroughly. Then, in the nonsurgical treatment of RCC, it could be an alternative adjuvant therapeutic option, especially in combination with other adjuvant therapies.

## Figures and Tables

**Figure 1:** The overview of phenotypes and proliferation rate of enhanced CIK cells and conventional CIK cells. (a) The representative data of flow cytometry. (b) The histogram showed quantified results of CD3^+^, CD3^+^CD4^+^, CD3^+^CD8^+^, and CD3^+^CD56^+^ cells in cultured enhanced CIK cells, conventional CIK cells, and PBMC and expressed as the percentage in lymphocytes. (c) The proliferation rate of enhanced CIK cells and conventional CIK cells. Difference between enhanced CIK cells and controls was determined by Student's *t*-test. ^*∗∗*^*p* < 0.01,^*∗∗∗*^*p* < 0.001, and *n* = 10.

**Figure 2:** Cytotoxicities of enhanced CIK cells against RCC cells and nonkidney cells. (a) The cytotoxic effects of CIK cells on HEK-293 and ACHN at a ratio of 8 : 1, 16 : 1, 32 : 1, and 64 : 1 (CIK/target cell). CIK treatment was initiated 24 h after seeding the tumor cells in 96-well plates. Cell viability was assessed by the CCK-8 after 36 h of CIK treatment. Results were expressed as percentages of CCK8 absorbance with respect to the untreated control wells (mean ± S.D. of 3 independent experiments with 3 wells each). Meanwhile, four nonkidney cell lines including SPC-A-1, HCT-116, BGC 823, and BEL 7404 were also studied for control. (b–d) The levels of granzyme B, perforin, TNF-*α*, and IFN-*γ* in supernate from ACHN cells or HEK-293 incubated with CIK cells. ^*∗*^*p* < 0.05, ^*∗∗*^*p* < 0.01,  and ^*∗∗∗*^*p* < 0.001 as compared with untreated control wells or CIK alone wells by Student's *t*-tests.

**Figure 3:** Scanning electron micrographs of ACHN cells treated with enhanced CIK cells. Green arrow: CIK cells; red arrow: ACHN cells. (a) 2500x magnification. (b) 5000x magnification. (c) 14000x magnification. (d) 30000x magnification.

**Figure 4:** Effects of enhanced CIK on nude mice model of xenograft. Mice were injected subcutaneously with ACHN cells 14 days before CIK treatment. Then, mice were randomly divided into four groups and administrated with CIK and PBS as control through intravenous injection or intratumoral injection. (a) The tumors were dissected from the mice and photographed. (b) All tumors collected from the back of each mouse were weighed. (c) The body weight of each mouse was monitored during the treatments. No difference was observed on 0 day and 35 days. (d–f) The effects of CIK treatments on the levels of granzyme B, perforin, and IFN-*γ* in serum obtained from mice after 21 days of treatments were analyzed by ELISA. ^*∗*^*p* < 0.05 CIK treatment group vs. control group (Student's *t*-test). The data are represented mean ± S.E.M. of 9 tumors.

**Figure 5:** The immunofluorescence staining of tumors collected from different treatment groups. (a) The representative photos of immunostaining of Ki67, TUNEL, and (b) CD3. (c) The histograms showed quantified results of positive-stained cells and expressed as percentage of control. *n* = 9, mean ＋ S.E.M., ^*∗*^*p* < 0.05, ^*∗∗*^*p* < 0.01,  and ^*∗∗∗*^*p* < 0.001, when compared with the PBS group vs. CIK group, by Student's *t*-test. Scale bars: 20 *μ*m.

**Figure 6:** Prognosis of patients in the enhanced CIK treatment group and control group. (a) Progression-free survival (PFS) and (b) overall survival (OS) were calculated by Kaplan–Meier analysis. Differences between the treatment group and control group were compared using the logRank test. (c) The representative CT scan images of lung metastases in RCC patients after CIK cells treatment. Case 1: a patient of RCC with lung metastasis at the beginning of follow-up, whose lung metastasis developed slowly during the 60 months follow-up period and no more metastatic lesion was observed. Case 2: a patient of RCC with lung metastasis at the beginning of follow-up, and the lung metastasis did not develop obviously in 18 months.

**Table 1:** The demographics and clinical characteristics of patients in the CIK group.

	Age/sex^*∗*^	TNM^*∗∗*^	Location of metastases	CIK cycles	Disease state after CIK cell treatment	Disease state by the end of follow-up	PFS (month)	OS (month)^*∗∗∗*^
Case 1	54/M	T1N0M0		5	CR	CR	60	60
Case 2	28/M	T2N0M0		4	CR	CR	60	60
Case 3	80/F	T1N0M0		4	CR	CR	21	34
Case 4	73/F	T1N1M0	Renal hilar lymph node	4	PR	SD	22	35
Case 5	48/F	T2N1M0	Renal hilar lymph node	5	PR	SD	36	60
Case 6	59/M	T2N0M0		5	PR	PD	10	16
Case 7	59/M	T2N0M0		3	CR	CR	32	32
Case 8	46/M	T1N0M1	Lung	4	PR	SD	36	60
Case 9	49/F	T2N0M0		2	CR	SD	21	45
Case 10	72/M	T2N0M1	Lung	4	PR	PD	11	30
Case 11	74/M	T2N0M0		5	CR	CR	38	60

CIK cycles: each cycle included 3 CIK infusions in 1 week and followed by a three-week rest. CR: complete response; PR: partial responses; SD: stable disease; PD: progressive disease.

**Table 2:** The demographics and clinical characteristics of patients in the control group.

	Age/sex^*∗*^	TNM^*∗∗*^	Location of metastases	Adjuvant therapy	Disease state at the beginning of the follow-up	Disease state by the end of the follow-up	PFS (month)	OS (month)^*∗∗∗*^
Case 1	47/M	T1N0M0			CR	CR	11	11
Case 2	70/M	T2N0M0			CR	PD	23	28
Case 3	49/M	T2N1M0	Renal hilar lymph node	IL-2 + IFN-*α*	PR	SD	21	29
Case 4	67/F	T1N0M0			CR	SD	31	41
Case 5	56/M	T2N0M0			CR	SD	18	32
Case 6	59/M	T2N1M1	Renal hilar lymph node&lung	IL-2 + IFN-*α*	PR	PD	6	15
Case 7	65/F	T2N0M0			CR	SD	23	45
Case 8	47/M	T1N0M0			CR	CR	52	52
Case 9	73/M	T2N0M0			CR	PD	11	21

CR: complete response; PR: partial response; SD: stable disease; PD: progressive disease. ^*∗*^Age: CIK: 58.36 ± 4.673; control: 59.22 ± 3.361; *p*=0.8880; sex: no difference between two groups (*p*=0.6424, Fisher's exact test). ^*∗∗*^TNM: no difference between two groups (*p*=0.5568, Mann–Whitney test). ^*∗∗∗*^The median survival of the CIK group and the control group was 45 months and 29 months.

## Data Availability

The data used to support the findings of this study are available from the corresponding author upon reasonable request.
